# Teaching Mode Based on Educational Big Data Mining and Digital Twins

This article has been retracted.

**DOI:** 10.1155/2022/9071944

**Published:** 2022-02-16

**Authors:** Xueyun Zhou, Xinling Wu

**Affiliations:** ^1^School of Engineering, Guangzhou College of Technology and Business, Guangzhou 510850, Guangdong, China; ^2^School of Computer Science, Guangdong Polytechnic Normal University, Guangzhou 510665, Guangdong, China

## Abstract

Data mining technology has gradually become an important data analysis and knowledge discovery technology widely used in many modern industries. Data mining is a technique to find its regularity from a large amount of data by analyzing each data. It mainly includes three steps: data preparation, regularity search, and regularity representation. Data preparation is to select the required data from relevant data sources and integrate them into a data set for data mining; regular search is to find out the regularity contained in the data set by a certain method; regular expression is to be as user-readable as possible. The way of understanding (such as visualization) will represent the found patterns. This research mainly discusses the improvement of teaching mode based on digital twin-based education big data mining. Through the research on the basic principles of data mining and digital twin technology, the student evaluation tool module based on digital twin and the relevant data analysis tool module of students based on digital twin education big data mining are developed. Data mining is carried out from the data of student performance, personal basic information, and evaluation information to find the correlation between various factors, find the hidden laws, and provide support for teaching decision-making. This paper also solves the problem of frequent communication with remote databases according to the characteristics of the database data required by students and improves the efficiency and scalability of education big data mining technology based on digital twins. The goal of the virtual interactive system of the digital twin-based CNC platform is to have both three-dimensional real-time monitoring and remote control functions based on a three-dimensional virtual CNC panel. This research integrates the three-dimensional real-time monitoring and remote control of the virtual interactive system, analyzes the system operation process, develops the system interface, and improves the system sub-functions; it builds an experimental environment, conducts example tests on various functions of the digital twin platform virtual interactive system, and performs virtual interactions system performance indicators are analyzed. 60% of students believe that their innovation ability has been improved after the implementation of the digital twin teaching model; 50% of students believe that their self-evaluation ability has been improved. Applying digital twin's educational big data mining to student information management, university teaching evaluation, student performance analysis, and examination system, it has played a very good guiding role in improving the level of school teaching management.

## 1. Introduction

In the modern higher education management, the level of informatization has been improved year by year. With the widespread use of campus cards and the accumulation of data from major business systems over the years, a campus big data environment has been formed. It is mainly reflected in the characteristics of large-scale, multi-type, high-speed, and low-density value of student data. How to effectively mine student behavior data has become an important content to improve the level of student work informatization management. The data mining education model not only makes up for the shortcomings of face-to-face education and single online education in the past, but is also consistent with modern education reforms. In the information age, educators must break traditional education concepts, explore new education models and methods, promote education and education reform, improve education and education quality, and promote students to develop in a better direction with the help of information technology.

By building a student behavior big data analysis system, it analyzes and processes the behavior characteristics of students in school, and applies it to the identification of students with financial difficulties in the school's student financial aid center. Through the reliability of massive data mining and the scientific nature of related algorithms, it changes the original mode of identifying work for students with financial difficulties from families, and implements the goal of improving the informatization of college students' work. The data mining education model mainly integrates online learning and offline learning through high-quality educational resources and intelligent learning platforms. In the process of mixed teaching, learners can not only communicate with classmates, but also communicate online at any time through the Internet. At the same time, students with fast learning progress can gain knowledge in advance through online learning, and students with slow learning progress can use network resources to further confirm and integrate knowledge to meet their learning needs.

The progress of virtual simulation resource construction urgently needs to be improved, the education system lacks top-level design, and the system construction standards are not unified. Schleich et al. believe that digitization of manufacturing industry promotes the application of complex virtual product model (called digital twin model) in all stages of product realization [1]. Li et al. believe that current airframe health monitoring often relies on deterministic physical models and ground inspections. He uses the concept of dynamic Bayesian networks. Dynamic Bayesian networks integrate physical models and various sources of contingent (random) and cognitive (lack of knowledge) uncertainty in crack propagation prediction [2]. Zhang et al. believe that new national advanced manufacturing strategies such as Industry 4.0, Industrial Internet and Made in China 2025 are introduced to realize intelligent manufacturing, and the number of new workshops in developed and developing countries keeps increasing. Under personalized design requirements, more realistic virtual models reflect the real world of manufacturing workshops, which is crucial to bridging the gap between design and operation [3]. Seay believes that for a critical infrastructure such as the national grid, the delay between identifying a cyber attack and deploying defenses can be disastrous. ORNL scientists are working to solve this problem with a platform called “digital twinning,” which provides real-time simulations of the grid so that system distortions can be identified almost immediately. The grid is often called the largest machine in the world. It is a complex and interdependent network consisting of power generation, transmission lines for long-distance transmission of power, substations for lowering the voltage of public utility systems, distribution lines connecting communities, and equipment for converting power for customers [4]. Fei et al. believe that digital twin (DT) is one of the most promising enabling technologies for intelligent manufacturing and Industry 4.0. The importance of DTs is increasingly recognized by academia and industry. It has been nearly 15 years since the concept of DT was first proposed. To date, many DT applications have been successfully applied in different industries, including product design, manufacturing, forecasting, and health management. However, there has not been a review of DT applications in industry. In order to understand the development and application of DTs in industry, he comprehensively reviewed the DT research status of key components of DTs, the development status of DTs, and the main application of DTs in industry. He also outlined current challenges and some possible directions for future work [5]. Tao et al. consider digital twinning to be a new and rapidly developing technology for connecting the physical and virtual worlds, which has recently attracted wide attention worldwide. This paper presents a new product design method based on digital twin method. First, the development of product design is briefly introduced. Then the framework of digital Twin driven Product Design (DTPD) is proposed and analyzed. A case is provided to illustrate the application of the proposed DTPD method [6]. Lydon et al. believes that new and refurbished buildings will require significant improvements in energy performance according to Swiss and EU targets for 2050. The construction industry, however, has a poor record of improving productivity and efficiency. As other industries have demonstrated, digital approaches can reduce product development time and costs by using numerical simulations to reduce prototyping. In addition, digital twin is an extensive computational model of a product that is planned to be improved over its life cycle by leveraging operational data. He presents coupled simulation of thermal design of heating and cooling systems integrated with lightweight roof structures. The shape of the concrete roof structure is optimized to provide a low-energy building element that is thermally activated to provide space conditioning from a renewable source of heat. This work focuses on modeling methods used in the energy sector to support the development of digital twins of multifunctional building elements [7]. Virtual models can predict, estimate, and analyze dynamic changes by understanding the state of physical entities through perceptual data. The physical object responds to the optimization in the simulation. Digital twinning can optimize the whole teaching process through the network-physical closed loop.

Today, with the rapid development of information technology, the development of scientific theories has brought about the rapid progress of science and technology [8, 9]. The progress of science and technology has an impact on the field of education all the time, and changes the way of education transmission. The promotion and dissemination of resources has played a role in fueling the flames, benefiting more and more people. The online virtual simulation teaching experiment system designed and implemented in this article follows the principle of “combining virtual reality, complementing each other, and realizing reality without vitality.” It actively explores the complementary advantages of various types of experiments in the experimental teaching design, combining virtual simulation, remote experiment, and optimized combination of physical experiments. It analyzes and evaluates the problems of low student performance, almost zero communication between teachers and students, single learning style, and long feedback period in the digital twin virtual teaching model, and proposes corresponding solutions. It combines the analysis and evaluation results to design the corresponding virtual teaching interaction center, and completes the development, testing, and evaluation of the entire virtual interaction center, and provides a decision-making reference for relevant education departments.

## 2. Teaching Mode Improvement Research Methods

### 2.1. Virtual Simulation Teaching Platform

Digital twin platform can be divided into online learning feature analysis technology and virtual-real teaching space fusion analysis technology. Through the deep integration, mapping, and mirroring between “online teaching” and “online learning,” it can inject new digital productivity into online immersive teaching [10]. First, deploy the developed experimental project to the business server. The uplink of the business server communicates with the user's client to transmit the user's operating parameters and the experimental data returned by the business server; the downlink communicates with the network management server, used to transmit the signaling of the service server and the experimental result data returned by the network management server. Second, the network management server regularly collects the status information of the registered LTE base stations through the heartbeat mechanism, and maintains the communication link with the base stations in the alive state; and through the connected computer that controls the mobile phone, it controls the switch of the mobile phone. Third, after the mobile phone is turned on, it connects to the LTE base station with the strongest signal around to establish a network channel. Remote users can select experimental items through the client computer and perform experimental control, including the configuration of base station parameters, adjustment of signal strength, initiating mobile Internet services, intercepting communication signaling, and other functions. The virtual simulation teaching platform is shown in Figure 1.

### 2.2. Three-Dimensional Digital Twin Podium Design

The combination of real-time modeling technology and virtual-real fusion technology, mainly through big data analysis, mining and modeling technology, carries out association rule analysis based on various algorithms on the association between virtual and real teaching spaces, so as to deeply analyze the relationship between virtual and real teaching spaces, and around the association, and then promote the integration of virtual and real teaching space.

The development of virtual platform interactive technology of 3D digital twin machine tool and multimedia blackboard control instructions is the basis of remote control technology of 3D virtual numerical control platform. By studying the interactive technology of the virtual CNC platform, it is possible to operate the virtual three-dimensional CNC platform to send commands. The development of immersive teaching control instructions can directly operate the multimedia blackboard. Coupling the interactive commands of the 3D virtual control platform with the control commands of immersive teaching can realize the remote control of the multimedia blackboard. After the virtual platform interactive technology is implemented, the digital twin teaching class needs to be equipped with a virtual numerical control platform. The three-dimensional digital twin teaching class corresponds to the virtual numerical control platform one-to-one, and the multimedia blackboard is remotely controlled through the virtual numerical control platform. As the control equipment of 3D digital twin teaching, the virtual numerical control platform has two main functions. First of all, the virtual numerical control platform can directly send debugging instructions to the 3D digital twin teaching terminal, which can simulate the teaching explanation process and adjust the key content of teaching to verify whether the 3D twin teaching has qualified performance. Then, the virtual numerical control platform can send control instructions to the multimedia server, and the multimedia server parses the control instructions into corresponding operation instructions. According to the different immersive teaching, the multimedia server sends different operation instructions to realize the remote control of the multimedia blackboard.

### 2.3. Main Interface of the Virtual Interactive System

The digital twin podium is a real-time dynamic mapping of the real online teaching space. Therefore, the real-time acquisition, transmission, and dynamic update of data are of great significance to it. The main interface of the virtual interactive system is mainly divided into the real-time monitoring area of the center podium and the surrounding chart menu bar area [11]. At the top of the system, there is a more detailed sub-menu bar and real-time display of the current frame number of the system. The chart area on the left shows the exact position of the current platform, the number of people online in real time, the current teaching code program, and the layout of the lecture content in turn. Client users can either watch the lecture process of the podium in real time through virtual roaming, or check the accurate information of the podium through the menu bar. In addition to the main interface, you can view other information of the CNC platform and class through the menu bar. The menu bar provides the entire class layout diagram, and the client operator can view the entire class status through the class layout diagram, understand the distribution of the platform, and prepare for the three-dimensional virtual roaming. Or it can select the multimedia file that needs to be transferred from the client, and then send it by the virtual numerical control panel. Hiding the sub-functions of the virtual interactive system through the sub-menu can provide the client operator with a better sense of immersion.

Divide the projection interval *T* on the *Y*-axis into *k* equally, then the length of each sub-interval is [12]

(1) $$\begin{array}{c} l=\frac{F_{x\max}-F_{x\min}}{k}. \end{array}$$

The points of the subset constitute the vertex subset *S*_*D*_ [13]:

(2) $$\begin{array}{c} S_{D}=\left(x,y,z\right)|F_{x\min}+\chi +f\left(x+1\right). \end{array}$$

The mean value of the three-dimensional coordinate vertex distribution *J* [14]:

(3) $$\begin{array}{c} J=\frac{1}{3M}\sum_{i=1}^{m}\left(p+q+r\right). \end{array}$$

The mean value of the peripheral vertex set can be obtained, and the covariance matrix *C* can be calculated [15]:

(4) $$\begin{array}{c} C=\frac{1}{3\text{m}}\sum_{i=1}^{m}\left(p_{1}p_{2}+q_{1}q_{2}+r\right). \end{array}$$

*C* is a symmetric matrix, and its eigenvectors *d*_1_, *d*_2_, and *d*_3_ are perpendicular to each other, and the three eigenvectors are unitized [16]:

(5) $$\begin{array}{c} d_{1}=\frac{d_{1}^{\prime }}{\left|d_{1}\right|},\\ d_{2}=\frac{d_{2}}{\left|d_{2}\right|},\\ d_{3}=\frac{d_{3}}{\left|d_{3}\right|}. \end{array}$$

### 2.4. Network Communication Module Design

The network communication module is mainly realized through the Socket Channel Server and Socket Channel classes. The module is mainly divided into four parts: message server, message receiver, message parser, and message type registration. The network connection between the interactive teaching system and the teacher server is realized through the XmlClient class. XmlClient needs to configure the IP address and listening port number of the teacher server. If the connection is successful, then XmlClient will add the connected Socket to the connection list for subsequent data Receive and send. All interactive messages in the interactive teaching system are extended from the XmlMsg class, and applications can flexibly configure new message types by inheriting from this class. XmlMsgHandler is the corresponding message parsing class that matches with XmlMsg. All message types on the mobile terminal of the interactive teaching system need to be registered in XmlMsgFactory. In addition to actively connecting with the teacher server, the mobile terminal of the interactive teaching system can also establish an XML conversation service by using XmlServer. The XmlServer class can monitor the network and add the clients connected to it into the connection list.

### 2.5. Platform User Demand Discovery Function Design Based on Big Data Technology

1. Platform users conduct learning activities and obtain portraits of current learning users. Platform users conduct learning activities through interaction with related applications. When platform users have a demand for teaching resources, they will conduct data queries. The traditional information retrieval process is to match the user's query set *Q* with teaching resources *U* to obtain teaching resources. In order to realize the perception of user needs, first collect the information of each dimension of the user portrait at the current time *t* through the application and its events such as user records, workflows, and learning tasks related to learning activities. The ontology semantic description forms the current learning user portrait.
2. User portrait matching is done, perceiving the demand for teaching resources. Calculate the similarity between the learning user portrait at the current time *t* and the historical application user portrait in the teaching resources of the integrated application user portrait, and through the process of demand discovery, demand screening and demand sorting, combined with platform user query conditions, the user's demand results are obtained.
3. Optimize teaching resources and add teaching resources integrating user portraits. The results of the teaching resources required by the platform users are fed back to the users. The users select and evaluate the teaching resource sets pushed by the system, or re-search and query the teaching resources, and use the learning activities to obtain the teaching resource application results, and compare them with the current teaching resources. They learn the integration of user portraits and form teaching resources corresponding to new user portraits. The realization process of user requirement discovery is shown in Figure 2.

Identify and obtain direct user profile information. When platform users perform learning activities in order to complete corresponding learning tasks, the platform user's personnel identification, teaching background, and learning task identification indicate that it belongs to the direct acquisition of information.

Association defines user portrait information. Obtain the historical records of platform users through the association with the teaching resource system, including participating tasks, learning achievements, teaching resources concerned, retrieval data, and resource evaluation. Among them, manual semi-supervision and process management are required, which can infer the class where the platform user is located, the portrait of other users in the class, etc., so as to obtain a more comprehensive user portrait.

In the guest user portrait model tree UC2, the corresponding node is *U*′, and the similarity calculation formula of the two nodes is [17]

(6) $$\begin{array}{c} \text{sim}\left(U,U^{\prime }\right)=\sum_{m=1}^{n}w*\text{sim}Q\left(U,U^{\prime }\right), \end{array}$$

where sim(*U*, *U*′) represents the node *U* and the corresponding node *U*′ [18].

The formula for calculating the similarity of single-valued character attributes is [19]

(7) $$\begin{array}{c} \text{sim}P\left(c_{1},c_{2}\right)=\left\{\begin{array}{cc} 1, & c_{1}\cdot \text{value}=c_{2}\cdot \text{value},\\ 0, & \text{other.} \end{array}\right. \end{array}$$

For two different single-valued numerical attributes similarity:

(8) $$\begin{array}{c} \text{sim}P\left(n_{1},n_{2}\right)=\frac{\left\|n_{1}-n_{2}\right\|}{\left|n_{1}\right|}. \end{array}$$

The similarity calculation of single-valued object attributes is equivalent to the nested calculation between user portrait elements [20]:

(9) $$\begin{array}{c} \text{sim}\left(o_{1},o_{2}\right)=\sum_{i=1}^{n}w_{j}\cdot \text{sim}p\left(o_{1},o_{2}\right). \end{array}$$

The similarity calculation method in the research process is [21]

(10) $$\begin{array}{c} \text{sim}\left(s,p\right)=\max\left(\text{sim}\left(s,s_{i}\right)|s\in p\right). \end{array}$$

Use |PS| to denote the number of elements in the set, and the calculation formula for the similarity between sets is [22]

(11) $$\begin{array}{c} \text{sim}\left(p_{1},p_{2}\right)=\frac{\sum \text{sim}\left(s,PS_{1}\right)+\sum \text{sim}\left(s,PS_{2}\right)}{PS_{1}+PS_{2}}. \end{array}$$

### 2.6. Specific Content of the Learning Evaluation Model for Digital Twin Teaching

Before the start of the course, first evaluate the students' learning goals. The purpose of evaluation is to determine whether the students' goals are reasonable, help students sort out their learning goals, and provide a good foundation and start for students' follow-up learning. At the input evaluation level, there are two aspects: the teacher's input and the student's input. The teacher's input includes the design and implementation of the mixed teaching model, and the establishment of a digital twin online learning platform.

The input of students mainly includes the emotional and attitude input of students in the learning process. This research mainly evaluates students. Therefore, only the input of students is selected as the main research content of input evaluation.

In process evaluation, the comprehensive ability of students is regarded as the main content of the evaluation. Teachers use the online learning platform to implement blended teaching, observe and analyze the learning behavior of students in the process of learning, and record and analyze the performance of students in activities and events.

In terms of achievement evaluation, the study effect of students is taken as the main research content, mainly to evaluate students' mastery of basic professional knowledge. Teachers learn the basic knowledge of students through various forms such as daily homework, group homework, individual independent homework, and final exams. The effect is comprehensively evaluated.

As a group, upload the work to the digital twin teaching platform. Groups can browse each other's works and evaluate other groups, and the scale for group evaluation will be uploaded to the platform by the teacher in advance. The component evaluation scale is shown in Table 1.

Teachers evaluate the students' personal assignments uploaded to the digital twin teaching platform, and score the students' daily assignments based on the personal assignment evaluation scale. The scale is also an important basis for evaluating students' learning effect and comprehensive ability. The personal work evaluation scale is shown in Table 2.

A general summary of the teaching resources that platform users need to query [23]:

(12) $$\begin{array}{c} C\left(QC\right)=\overset{m}{\underset{i=1}{U}}\left(mk\left(ef\right)\right). \end{array}$$

The result set of educational resources formed after query and screening is as follows [24]:

(13) $$\begin{array}{c} MK\left(F\right)=\overset{m}{\underset{i=1}{U}}\left(mk\left(ef\right)\right),\;m>0,\\ MK=\left(MK_{1},MK_{2},\ldots ,MK_{n}\right). \end{array}$$

The big data demand results obtained are [25]

(14) $$\begin{array}{c} W\left(MK\right)=\left(∐W_{1}\left(MK_{1}\right),∐W_{2}\left(MK_{2}\right),\ldots ,∐W_{N}\left(MK_{N}\right)\right). \end{array}$$

The set of teaching resource requirements is [26]

(15) $$\begin{array}{c} MK_{QC}=QC_{P}\cup QC_{T}\cup QC_{O},\\ MK=MK_{QC}-MK_{ef}. \end{array}$$

Digital twin learning satisfaction *P*_*Q*_ can be expressed as [27]

(16) $$\begin{array}{c} P_{Q}=P_{R}\cdot {\text{sim}}_{R}+P_{R}\cdot {\text{sim}}_{R}+P_{P}\cdot {\text{sim}}_{P}+P_{O}\cdot {\text{sim}}_{O}. \end{array}$$

The vector index of different learning objects is [28]

(17) $$\begin{array}{c} \overset{⟶}{QC}=\left\{T_{1},T_{2},T_{3},T_{R}\right\}. \end{array}$$

The query vector of the learning process can be expressed as [29]

(18) $$\begin{array}{c} \overset{⟶}{QC_{g}}=\left\{T_{1},T_{2},T_{2}-T_{3},T_{3}-T_{R}\right\}. \end{array}$$

## 3. Results of Educational Big Data Mining on the Improvement of Teaching Mode

The average score of the three rounds of action research is on the rise. Due to the step-by-step improvement of the teaching design, the number of people who get full marks has increased sharply. The higher degree of completion of classroom tasks also proves the rationality of teaching design and the improvement of teaching effect. The effect of teaching design is shown in Figure 3.

The sample students' learning objective evaluation grade scores are shown in Table 3.

According to the submission of students' works, the evaluation of students is shown in Table 4.

Calculate the average scores of comfort, adaptability, interactivity, sense of interest, and sense of immersion in the evaluation dimensions of students in the three classes of ABC. The comparison of each item is shown in Figure 4. It can be seen that with the update of the teaching design, the average scores of comfort, adaptability, interactivity, sense of interest, and immersion have shown an upward trend. Some have a large increasing trend, and some have a small increasing trend with a relatively high score.

In the course of teaching practice, the number of students who actively participated in the three rounds of action research was counted. The specific data are shown in Table 5. The first round of action research is the first time that digital twin teaching equipment has been brought to Class A classrooms. The number of students in Class A who are willing to try is relatively small. In the next two rounds of action research, there are more people willing to participate in the digital twin teaching experience. After the first round of action research, taking into account the students' unfamiliarity with the new technology, the students will be specially trained in the simple operation skills of digital twin teaching before class. The students in the class behave more positively, and the classroom atmosphere is better.

Achievement rate is an intuitive standard that reflects the realization of teaching goals. In the process of teaching practice, the number of students who have completed the immersive exploration of digital twin teaching is deliberately counted. The specific data are shown in Table 6. Among them, only five students in Class A successfully completed the digital twin teaching immersion exploration, which indirectly shows that these students have a particularly strong ability to accept new things. The achievement rate of Class B and Class C is relatively high, which is partly related to the timely adjustment of teaching design. I feel the charm of new technology more, and it is also an affirmation of the introduction of virtual reality technology into the classroom.

The performance test aims to test the performance of the mobile terminal of the interactive online teaching system when interacting with the teacher terminal. The timely response of interactive data has a great impact on the interactive experience, which needs to be paid attention to. The test is divided into non-optimized and optimized. The main test is the round-trip delay of interactive data between teacher and student equipment. Taking into account the frequency of interaction, the test mainly uses interactive whiteboard tools as the test target. Compared with the synchronization of courseware playback, the amount of synchronized data of the interactive whiteboard is larger, which can better explain the actual situation. First, consider the interactive data transmission round-trip time between the teacher and the student without closing the digital twin platform, as shown in Figure 5.

After closing the digital twin platform, the round-trip time of interactive data transmission between the teacher and the student is shown in Figure 6.

When the students answer the questions synchronously, the interactive teaching application has a small overhead, kept within 10%, which can be applied to more complex situations. The cost of interactive teaching applications is shown in Figure 7.

Among the students surveyed, more than 80% of students believe that their problem-solving skills have been improved after the implementation of the digital twin teaching model; more than 70% of students believe that their project practice skills, teamwork skills, and language expression skills have been improved; 60% of students believe that their innovation ability has been improved after the implementation of the digital twin teaching model; and 50% of students believe that their self-evaluation ability has been improved. The student ability evaluation is shown in Figure 8.

Students A and B have relatively high evaluation scores in terms of learning objectives, indicating that they have a clearer understanding of the course content before learning, but their learning attitude is at an intermediate level compared to other students and needs to be further improved. In terms of comprehensive ability and learning effect evaluation, further improvement is needed from the overall level. The overall level evaluation is shown in Figure 9.

## 4. Discussion

The teaching management department of colleges and universities needs to supervise and count the teaching quality of teachers, which requires the establishment of a scientific teaching evaluation system to carry out statistics and analysis of the status quo in the teaching quality process. Students are the objects of teachers' teaching courses, and they are also the key to improving teaching quality. Therefore, students' evaluation of teachers' classroom teaching has a very objective and realistic value. At present, many colleges and universities in China have adopted a teaching evaluation system based on student evaluation, teacher mutual evaluation, and self-evaluation. After many years of evaluation information feedback, many colleges and universities have accumulated a large amount of teaching evaluation data. The statistical results of the data serve as the basic basis for teachers' evaluation of awards, excellence, and job titles, and play the basic role of teaching evaluation data. However, with the development of information technology, simple data statistics can no longer meet the needs of university teaching management departments, because simple data statistics cannot find the potential teaching information that exists within the data, and more valuable data may be ignored by us. How to scientifically, rationally, and effectively use years of teaching evaluation data to guide teachers' teaching and improve teaching quality has become a very meaningful research topic.

Digital twin technology provides the architectural guidance of networked control and the direction of cyber-physical system realization. With the help of digital twin technology based on informatization and networking, the development of the system can take advantage of the computing power and information fusion capabilities of the entire industrial network to give play to the advantages of new machine learning algorithms and data-driven algorithms. The leveling control and anomaly detection algorithms, as well as the realization of related algorithms, are further studied and improved, combining information from different fields to achieve intelligent and networked control.

Subjective weight distribution requires the induction and extraction of human experience before the algorithm is executed. Although human experience has a strong individual dominance, the experience accumulated over the years cannot be replaced by any tool for induction and summary, and the value of human experience cannot be underestimated. The weight distribution based on objective conditions is actually the weight distribution based on objective data. It mainly analyzes the actual data that actually exists according to a certain algorithm, and finally obtains the weight value of the indicator based on the objective data. This method is based on objective facts. In order to analyze the data based on the facts, the results must be consistent with the objective facts. The objective weight determination method has a strong ability to persuade the data, and the results are reasonable. In the era of big data today, in the era of rapid economic and technological development in China, our focus has slowly shifted from food, clothing, housing, and transportation to education issues. We are in line with the world, and we want to accept better and more cutting-edge technologies. But what everyone can do in today's society is to perform their duties with full responsibility and help improve the way we are educated and the environment. This requires each of our students to face each answer sheet of teaching evaluation with a positive and serious attitude, and to attach their own opinions on classroom teaching after completing the selection of teaching evaluation indicators. At the same time, it is also required that educators in our schools and even the country can use the existing technical conditions to systematically analyze the real and effective teaching evaluation data, and combine the results of teaching experience and mathematical statistics to make an adjustment, an improvement, so that all enjoy the power that technology brings to education.

Three-dimensional real-time monitoring based on digital twins requires high enough real-time data. Remote monitoring in digital twins is the basis of course early warning and remote control. In the past, the delay of monitoring systems is often at the second level, which cannot meet the requirements of remote real-time monitoring in digital twins. Three-dimensional real-time monitoring based on digital twins requires the graphics processing speed to be fast enough. The essence of the digital twin model of the virtual interactive class is the superposition of multi-dimensional elements in computer graphics. The digital twin model of the virtual interactive class is highly complex, the monitoring scene modeling is huge, and the data update speed is very fast.

The database is the basis of the entire system, and its quality is directly related to the realization of the system. In traditional education management and education concepts, education statisticians must meet the requirements of data mining, use different spreadsheets to handle the traditional data management of the new student data classification system, and process the data. This is a new design requirement of the database, which requires mutual conversion and spreadsheet functions. Due to the realization of global information resource sharing, the surge of information, and the improvement of information demand, traditional information extraction methods cannot meet the practical needs, so data mining technology is proposed. Data mining technology is used to extract and analyze large amounts of data to find hidden clues and provide a more valuable basis for further decision-making. Data mining is based on the database for research. The ultimate goal of the researcher is to combine the database and data mining to make the final decision. In today's high-tech development, the scope of application of data mining is becoming wider and wider. It is not only suitable for university management, but also promotes the further reform, improvement, and development of school management, and also provides a good way for managers to make correct decisions. The educational management methods of basic schools have also been improved [30].

Generating a data warehouse is mainly about interface design and data loading interface design to ensure that the data extraction, transformation, and integration from the operational environment to the data warehouse can be completed and accurately completed with flexibility and variability. When loading data, ensure the order of data loading, filter invalid and wrong data, and manage data granularity. Design the interface from the database system to the data warehouse system to complete data purification and integration other than data extraction. The design of a data warehouse is an iterative process. As the process progresses, user needs are constantly clarified and the data that users really need are determined.

The national plan is based on education, and education is not a trivial matter. Teaching is different from business. Because there is no huge profit margin and long input-output time period, the application of high-tech in the teaching field is relatively backward and low in effectiveness. Appropriate methods are adopted to attract more scholars to use high-tech to transform teaching. It is a new problem facing the education system. Perform correlation analysis on students' personal basic information and results, various evaluation indicators, and project information that users are interested in, and look for the impact of students' personal basic conditions on student performance and evaluation indicators, as well as the interrelationship between results and various evaluation indicators. Data mining techniques are used to find the final result [31].

## 5. Conclusion

Although traditional face-to-face classroom teaching can effectively solve the above problems, it cannot meet the requirements of students in individualized learning and autonomous learning. In addition, traditional face-to-face teaching is mainly based on teachers, and students are in a passive position, which is not conducive to students' independence and innovation. The introduction of educational data mining technology into the digital campus system not only improves the scientific nature of education management, but also enhances the effectiveness of the digital construction of education. This system provides teachers and students with a digital twin virtual online interactive teaching platform that is easy to interact, manage, and operate. At present, the entire system has a large amount of data storage, including teacher data and student data. The education management information system only has simple query, statistics, and print functions for such a huge amount of data. If we can dig and analyze these data in depth, and discover some kind of internal connection, we will get some beneficial suggestive information. This article first made the overall design of the system, then designed the specific functions of the system, and then showed the experimental results of the system. The research in this field has certain potential, and the efficiency of digital twins in this article needs to be further improved.

## Figures and Tables

**Figure 1:** Virtual simulation teaching platform.

**Figure 2:** The realization process of user requirement discovery.

**Figure 3:** Teaching design effect.

**Figure 4:** Each comparison.

**Figure 5:** Interactive data transmission time between teacher and student without closing the digital twin platform.

**Figure 6:** After closing the digital twin platform, the interactive data transmission round-trip time between the teacher and the student.

**Figure 7:** The cost of interactive teaching applications.

**Figure 8:** Student ability evaluation.

**Figure 9:** Overall level evaluation.

**Table 1:** Component evaluation scale.

First-level index	Points	Secondary indicators	Points
Topic selection	10	Reasonable topic selection	10

Content	40	Completeness	25
		Innovation	15

Express display	25	Language expression	15
		Gallery	10

**Table 2:** Personal work evaluation scale.

Evaluation index	Grade			
	Weights	Excellent (80–100)	Pass (60–80)	Unqualified (0–60)
Accuracy	0.4	Correct	Basically correct	Confusion, error
Innovation	0.3	Ideas and insights	Lack of novelty	Nothing new
Organized	0.3	Clear logic	Basically ok	No logic

**Table 3:** The learning objective evaluation grade scores of the sample students.

Learning target situation	Grade	Grade-corresponding score
The learning objectives are clear and feasible	A	95
The learning objectives are clear and feasible	A	95
The learning objectives are clear and feasible	A	95
The learning objectives are clear, and the feasibility of the learning objectives needs to be improved	B	85
The learning objectives are clear, and the feasibility of the learning objectives needs to be improved	C	75

**Table 4:** Evaluation of students.

Student ID	Accuracy (0.3)	Completeness (0.2)	Innovation (0.2)	Organized (0.3)
A	100	95	80	85
B	90	90	85	80
C	85	85	95	90
D	85	90	80	85
E	90	85	85	80

**Table 5:** Number of students actively participating in the three rounds of action research.

Class	A	B	C
Total people	18	18	18
Number of active participants	8	15	17
Participation rate	44.44%	83.33%	94.44%

**Table 6:** Number of students who completed VR immersion exploration.

Class	A	B	C
Total people	18	18	18
Number of people reaching the target	5	12	17
Achievement rate	27.78%	66.67%	94.44%

## Data Availability

No data were used to support this study.
